The article "A New Mutation of the INSR Gene in a 13-Year-Old Girl with Severe Insulin Resistance Syndrome in China" was published in 2021. Journal: Biomed Res Int.

# A New Mutation of the INSR Gene in a 13-Year-Old Girl with Severe Insulin Resistance Syndrome in China

**DOI:** 10.1155/2021/8878149

**Published:** 2021-02-25

**Authors:** Jing Jin, Xinxin Liang, Jie Wei, Lingling Xu

**Affiliations:** Department of Endocrinology, Shenzhen Hospital, Southern Medical University, Shenzhen 518100, China

## Abstract

**Background:**

Mutations in insulin receptor genes can cause severe insulin resistance syndrome. Compared with Rabson-Mendenhall Syndrome and Donohue's Syndrome, type A insulin resistance syndrome is generally not serious. The main manifestations in woman with type A insulin resistance syndrome are hyperinsulinemia, insulin resistance, acanthosis nigricans, hyperandrogenism, and polycystic ovary. *Case Presentation*. A 13-year-old girl (Han nationality) visited the hospital due to hairiness and acanthosis nigricans. Further examination revealed severe hyperinsulinemia, insulin resistance, elevated blood glucose, hyperandrogenism, and polycystic ovary. Analysis of the insulin receptor gene by sequencing showed the presence of a nucleotide change in intron 7 (c. 1610+1G > A). The mutation was a splicing mutation, which can obviously affect the mRNA splicing of the insulin receptor and cause its function loss. The patient was finally diagnosed with type A insulin resistance syndrome. After 2 months of metformin treatment, the patient had spontaneous menstrual cramps and significantly improved acanthosis nigricans and sex hormones.

**Conclusion:**

We report for the first time a new splicing mutation on the insulin receptor gene at the 7th intron (c.1610+1G > A), which leads to type A insulin resistance syndrome. In clinically suspected patients with polycystic ovary syndrome, if there are extremely high blood levels of insulin in the blood, genetic testing should be performed to detect insulin receptor gene mutation of type A insulin resistance syndrome.

## 1. Introduction

Inherited insulin resistance syndrome refers to a class of diseases related to mutations in insulin, insulin receptor (INSR), and postreceptor genes [1]. INSR gene mutation is the most common one, causing type A insulin resistance syndrome or Rabson-Mendenhall Syndrome and Donohue's Syndrome [2]. The symptoms of type A insulin resistance syndrome are relatively mild. The diabetes of patients with this syndrome is generally not severe, and patients can survive to adulthood [3]. Type A insulin resistance syndrome is mainly manifested by severe insulin resistance, hyperinsulinemia, hyperandrogenism, and acanthosis nigricans. Thus, it is easy to be misdiagnosed as polycystic ovary syndrome [4]. Here, we described an adolescent female who was clinically suspected of polycystic ovary syndrome and finally confirmed as type A insulin resistance syndrome by genetic testing. Moreover, a new splicing mutation on the INSR gene at the 7th intron (c.1610+1G > A) was identified in this case.

The article "A New Mutation of the INSR Gene in a 13-Year-Old Girl with Severe Insulin Resistance Syndrome in China" was published in 2021. Journal: Biomed Res Int.

## 2. Case Report

A 13-year-old girl was admitted to our department because of hairiness and melanosis in skin folds. The patient was born with a birth weight of 3000 g. Her family history was unknown because she was adopted in infancy. The patient had similar growth and development to her peers and had no history of long-term medication. Two years ago, the patient began to have increased body hair, dense sexual hair, and a weight increase of about 5 kg. Skin pigmentation gradually appeared, the skin became dark, and there was no menstruation. A 75 g glucose tolerance test was performed in another hospital, which showed that fasting blood glucose was 4.42 mmol/L and 2-hour blood glucose was 15.37 mmol/L. Transrectal Color Doppler ultrasound of uterine annex showed suspicious polycystic changes in both ovaries. Physical examination showed the following: height 160 cm, weight 56.3 kg, BMI 21.99 kg/m^2^, increased body hair, dense sexual hair, and perineal sexual hair in a rhombic distribution. Ferriman-Gallwey Score was 25. The skin showed acanthosis-like changes. There was no acne or thyroid enlargement. Her pubertal development was Tanner grade IV, and bone age was 13 years. Liver and kidney functions, blood lipids, thyroid function, 17 hydroxyprogesterone, and electrolytes were normal. Cortisol rhythm was also normal (245.8 nmol/L at 8 am; 122.3 nmol/L at 4 pm; and 22.21 nmol/L at 12 am; 4.33 ng/mL of ACTH at 8 am). At 24 hours, urine free cortisol was 382.42 nmol (reference range 57.70-806.80) and dehydroepiandrosterone sulfate was 192.00 *μ*g/dL (reference range 35.0-430.0). Hormonal pattern cycle was as follows: follicle stimulating hormone (FSH)—6.74 mIU/mL; luteinizing hormone (LH)—16.84 mIU/mL; testosterone—0.89 ng/mL; estradiol—37.28 pg/mL; progesterone: 0.64 ng/mL; prolactin—11.93 ng/mL; and sex hormone-binding globulin—10.60 nmol/L. Upon reexamination, the fasting blood glucose was 4.41 mmol/L; the simultaneous fasting insulin was 106.9 *μ*U/mL; 2-hour postprandial blood glucose was 7.6 mmol/L, and the simultaneous postprandial insulin was more than 1000 *μ*U/mL. The clinical manifestations and laboratory diagnosis of this patient tend to be polycystic ovary syndrome, but this patient had higher insulin levels than those with polycystic ovary syndrome. However, the blood glucose did not increase significantly. Therefore, after obtaining the consent of patients and their families, we further performed genetic testing. The results showed that there was a mutation on the INSR gene (c. 1610+1G > A) (Figure 1). This mutation was a heterozygous splicing mutation, which may result in function loss of the INSR. This mutation is not reported before in the HGMD database nor found in any of the ESP6500siv2_ALL, dbSNP147, and Thousand Genome (1000g2015aug_ALL) databases. After being annotated by ANNOVAR [5], this mutation could significantly affect mRNA splicing. Therefore, the patient was diagnosed with type A insulin resistance syndrome. We recommended the patient to strengthen exercise and control diet. Metformin of 1.5 g/day was administrated for treatment. Two months later, the patient had spontaneous menstruation. The symptoms of acanthosis nigricans were improved obviously. Blood glucose levels and the ratio of LH/FSH were normal (Table 1). Insulin levels decreased but were still higher than normal levels. However, the testosterone level did not change obviously (Table 1). Unfortunately, the patient did not continue to be followed up in our hospital since then.

The article "A New Mutation of the INSR Gene in a 13-Year-Old Girl with Severe Insulin Resistance Syndrome in China" was published in 2021. Journal: Biomed Res Int.

## 3. Discussion

The human INSR gene is located on the autosome 19p13.2-13.3, with a total length of more than 170 kb and contains 22 exons and 21 introns. The exon 1-11 encodes the *α* subunit, and the exon 12-22 encodes the *β*-subunit [6]. The *α* unit is the part that binds to insulin and is located outside the cell, while the *β*-subunit is a transmembrane peptide chain whose intracellular domain contains tyrosine kinase activity [7]. The homozygous mutation of the *α* subunit is usually manifested as Donohue syndrome or Rabson-Mendenhall syndrome, which is clinically rare and has a very poor prognosis. *β*-Subunit mutations mostly lead to decrease or loss of tyrosine kinase activity, which is common in patients with type A insulin resistance syndrome [8, 9]. However, there are also homozygous mutations in the *α* subunit in patients with type A insulin resistance, and patients with Donohue syndrome or Rabson-Mendenhall syndrome can also be caused by mutations in the *β*-subunit [10, 11]. There are 132 pathogenic mutations in the INSR, most of which are missense and nonsense mutations (78%) and only 8 mutation sites are located in introns [12]. Longo et al. found that a patient with Donohue syndrome carried biallelic mutations, one of which was a splice donor junction in intron 13; but the mother who carried intron 13 mutation had normal phenotype, suggesting that the mutation of the intron may be recessive [13]. Magre et al. reported a case of a heterozygous mutation in intron 14 of the INSR gene in a patient with type A insulin resistance syndrome [14]. They further measured the mRNA level of the INSR gene and tested the function of the INSR and found that the mutation significantly reduced the number and function of the INSR. In this study, the patient who manifested as type A insulin resistance syndrome carried a new heterozygous splicing mutation at the intron 7 of INSR. However, it is still uncertain whether this mutation at the intron 7 of INSR can directly cause type A insulin resistance syndrome. Further investigation is needed.

The article "A New Mutation of the INSR Gene in a 13-Year-Old Girl with Severe Insulin Resistance Syndrome in China" was published in 2021. Journal: Biomed Res Int.

The clinical symptoms of type A insulin resistance syndrome are mainly caused by insulin resistance and hyperinsulinemia. Because these patients have defects in the function of their INSR, it has been proposed that the “toxic” effects of hyperinsulinemia may be mediated by receptor for homologous peptides such as IGF-1 [15]. In the early stage of the disease when the beta cells of the pancreas are normal, there may be compensatory increase in the proliferation of beta cells or their secretory function, resulting in an increased amount of insulin. Thus, the blood glucose level can be maintained relatively normal. Diabetes occurs when the function of pancreatic islet beta cells fails and the level of insulin decreases or its increases are not enough to compensate the blood glucose. For adolescent or childbearing women, there will be polycystic ovary syndrome and even infertility [16]. The related mechanisms are as follows: (1) direct stimulation of the ovaries to secrete androgens; (2) increase of luteinizing hormone-induced androgen secretion by inducing steroid hormone synthase; (3) increase of gonadotropin-releasing hormone pulse secretion, leading to ovarian dysfunction; (4) reduction of the synthesis of sex hormone binding globulin in the liver, resulting in increased free testosterone; and (5) promotion of the secretion of anti-Mullerian hormone, leading to midterm sinus follicle development retardation [17]. Elevated androgen levels lead to varying degrees of hairiness and virilization [18]. High-concentration insulin can bind to the INSRs or insulin-like growth factor-1 receptors remaining on the keratinocytes and dermal blasts of the neck, face, and armpits, forming acanthosis nigricans. When high-concentration insulin combines with receptors in other parts of the limb, it can cause pseudoacromegaly manifestations such as nail hypertrophy, forehead bulge, skin thickening, hand, and foot enlargement [19]. Interestingly, unlike patients with ordinary insulin resistance, the weight of patients with type A insulin resistance syndrome has not increased significantly [3].

## 4. Conclusions

In summary, type A insulin resistance syndrome is caused by mutations in the INSR gene. Gene mutations are widespread and can be located in the *α*- or *β*-subunits and in exons or introns in type A resistance syndrome. These mutations influence the synthesis of INSR protein and lead to severe insulin resistance. We have reported a new mutation site in the INSR gene, but whether this mutation will cause type A insulin resistance syndrome requires further testing. The current diagnosis of type A insulin resistance syndrome is mainly through clinical symptoms and genetic testing. For children and adolescent women who are not obese but have severe insulin resistance, irregular menstruation, hyperandrogenism, and acanthosis nigricans, gene screening should be performed for early detection and active intervention, which is also beneficial to future generations. However, due to the individual differences in gene mutations, the therapeutic effects are also very different. Controlling patients' metabolic disorders and active symptomatic management of complications are also important ways of treatment.

The article "A New Mutation of the INSR Gene in a 13-Year-Old Girl with Severe Insulin Resistance Syndrome in China" was published in 2021. Journal: Biomed Res Int.

## Figures and Tables

**Figure 1:** Sequencing results of mutation on the insulin receptor gene of patients. The arrow in the picture shows the mutation of c.1610+1G > A.

**Table 1:** Results of blood glucose, insulin, and sex hormones before and after treatment.

Items	FBG (mmol/L)	FINS (*μ*U/mL)	PBG (mmol/L)	PINS (*μ*U/mL)	LH (mIU/mL)	FSH (mIU/mL)	T (ng/mL)
Upon admission	4.41	106.9	7.6	>1000.00	16.84	6.74	0.89
2 months after treatment	4.37	78.4	5.59	634.1	7.74	5.02	0.83

FBG: fasting blood glucose; FINS: fasting serum insulin (reference range 2.6-24.9); PBG: postprandial blood glucose; PINS: postprandial serum insulin; LH: luteinizing hormone (reference range 2.4-12.6); FSH: follicle stimulating hormone (reference range 3.5-12.5); T: testosterone (reference range 0.025-0.268).

## Data Availability

The data that support the findings of this study are available on request from the corresponding author.
